# Herbal formula GAPT prevents beta amyloid deposition induced Ca^2+^/Calmodulin-dependent protein kinase II and Ca^2+^/Calmodulin-dependent protein phosphatase 2B imbalance in APPV717I mice

This article has been retracted.

**DOI:** 10.1186/s12906-016-1144-7

**Published:** 2016-06-01

**Authors:** Jing Shi, Xuekai Zhang, Long Yin, Mingqing Wei, Jingnian Ni, Ting Li, Pengwen Wang, Jinzhou Tian, Yongyan Wang

**Affiliations:** The 3rd Department of Neurology, Dongzhimen Hospital, Beijing University of Chinese Medicine, Beijing, 100700 China; Key Laboratory of Chinese Internal Medicine, Ministry of Education, Beijing University of Chinese Medicine, Beijing, China; Institute of Clinical Medicine, China Academy of Chinese Medical Sciences, Beijing, China

## Abstract

**Background:**

Synaptic dysfunction is one of the pathological characteristics of Alzheimer's disease (AD), which is directly related to the progressive decline of cognitive function. CaMKII and CaN have been found to play important roles in memory processes and synaptic transmission. So present study aimed to elucidate relationships between CaMKII, CaN and cognitive decline in APPV717I mice, and to reveal whether the cognitive improving effects of GAPT is conducted through rebalance CaMKII and CaN.

**Methods:**

Three-month-old-male APPV717I mice were randomly divided into ten groups (*n* = 12 per group) and received intragastrically administrated vehicle, donepezil or different doses of herbal formula GAPT for 8 or 4 months. Three-month-old male C57BL/6 J mice was set as vehicle control.

**Results:**

Immunohistochemistry analysis showed that there were CaMKII expression decrease in the CA1 region of APPV717I transgenic mice, while the CaMKII expression of donepezil or GAPT treated transgenic mice were all increased. And there were CaN expression increase in the brain cortex of APPV717I transgenic mice, while there were decrease of CaN expression in donepezil or GAPT treated transgenic group. Western blot analysis showed the similar expression pattern without significant difference.

**Conclusion:**

GAPT extract have showed effectiveness in activating the expression of CaMKII and inhibiting the expression of CaN either before or after the formation of amyloid plaques in the brain of APPV717I transgenic mice, which may in certain way alleviated neuron synaptic dysfunction in AD.

## Background

Dementia is estimated to affect as high as 24 million worldwide, and is predicted to double every 20 years through to 2040 [1]. As the leading cause of dementia, Alzheimer disease (AD) is clinically characterized by progressive decline in cognitive function, and pathologically characterized by neurofibrillary tangles, senile plaques and synaptic dysfunction. There are increasing researches on the correlation between synaptic loss and AD since the relationship was established initially [2]. Synapses is considered to be the earliest site of AD pathological change, and the rate of synaptic loss is directly related to the severity of the disease [3, 4]. While, synaptic transmission, with underlying phenomena like long term potentiation (LTP), has been proved to be a cellular model of learning process [5–8]. Among the molecules implicated in synaptic transmission, Ca^2+^/calmodulin (CaM)-dependent protein kinase II (CaMKII) and Ca^2+^/Calmodulin-dependent protein phosphatase 2B (calcineurin, CaN) have been found to play important roles in memory processes and neuronal degeneration [9–16]. CaMKII, a ubiquitous serine/threonine protein kinase, regulates biosynthesis & exocytosis of neurotransmitters,synaptic plasticity and many other cellular functions [9, 11, 12, 16–18]. It is highly expressed in the brain, especially in the hippocampal formation [19–22], with the characters of autophosphorylation and converting itself from the Ca^2+^-dependent form to the Ca^2+^-independent form [23]. And such increased autophosphorylation is essential for the long-lasting increase in synaptic efficacy following long-term potentiation (LTP) in the hippocampus [24]. On one hand, Genetic CaMKII gene disruption or CaMKII inhibitors blocking LTP were found in vivo or in vitro studies [25–27]. On the other hand, viral vector mediated expression of active CaMKII or active form of CaMKII injection increases α-amino-3-hydroxy-5-methyl-4-isoxazolepropionic acid receptor (AMPAR)-mediated synaptic transmission and occludes further induction of LTP [28–30].

Calcineurin (CaN), also known as protein phosphatase 2B (PP2B), is a calmodulin-dependent serine/threonine phosphatase physiologically activated by Ca^2+^. It is also highly expressed in the central nervous system [31] and responsible for the dephosphorylation of p-CaMKII. CaN is composed of a catalytic subunit (calcineurin A) and a tightly bound regulatory subunit (calcineurin B) [14, 15]. It has been intensely studied as a potential modulator of both memory processes and neuronal degeneration. However, there are still controversies about the relationship between CaN and cognitive decline. From one aspect, activation of CaN in aged rats is related with cognitive decline [32] and its inhibition improves memory performance in some normal aging rodents, as well as in some APP over expressing AD models [33–36]. From another aspect, CaN activity has been reported being reduced in the cortex of AD patients [37, 38]. Interestingly, recent researches have revealed the details behind the relationship between CaN and AD. There are evidences to suggest that Aβ induces different changes of CaN expression in neurons and astrocytes [39]. Its catalytic subunit, CaN A, is proteolytically activated in AD cortex by the degradation of an autoinhibitory domain [40], which is expressed in reactive astrocytes surrounding senile plaques [41]. It has been proposed that amyloid beta (Aβ)-induced perturbation of LTP potentially involves enhanced CaN activity, and the latter creates an imbalance between CaN and PKA activity, causing over activation of protein phosphatase 1 (PP1). While, PP1 acts as a regulator of the phosphorylation of CaMKII, and therefore, ultimately influences dephosphorylation of CaMKII (reviewed by [42]).

However, there are still not very clear on the relationships between CaMKII, CaN and cognitive decline in APPV717I mice. So this study aimed to elucidate their relationships and reveal whether the cognitive improving effects of GAPT is conducted through rebalance CaMKII and CaN.

GAPT, also called as GEPT in our previous papers, is a combination of herbal extracts, including eight active components pro rata of Ginsenoside from ginseng 4.4 %, Cistanche 17.3 %, Radix Rehmanniae 17.3 %, Polygala tenuifolia 13 %, Acorus tatarinowii 13 %, Radix Curcumae 13 %, Poria cocos 13 %, Salvia officinalis 9 % [43].

Owing to the kidney deficiency and phlegm turbid pathogenesis of AD, GAPT was made according to the therapeutic principle of reinforcing kidney Yang and reducing phlegm. That is Ginseng, Cistanche, Radix Rehmanniae and Poria cocos reinforcing kidney; while Acorus tatarinowii, Radix Curcumae, Salvia officinalis and Polygala tenuifolia reducing phlegm turbid. Previous studies indicated that GAPT extract can markedly improves learning and memory of AD rat models made from hippocampal injection of Aβ1-42 peptide or intravenous injection of Aβ1-40 peptide [44], and reduces the level of Aβ in APPV717I transgenic mice via inhibiting γ-secretase (presenilin-1) and promoting insulin degrading enzyme and neprilysin [43]. Moreover, GAPT also showed significant improvement on cognitive function in patients with amnestic mild cognitive impairment (aMCI), an intermediate stage between normal aging and the more serious decline of AD, consistently across different cognitive scales in a 24-week preliminary clinical study [45]. While, the mechanisms behind synaptic protection effects of GAPT is still not well understood. This study therefore aimed to reveal the influences of GAPT in the balance of CaMKII and CaN.

## Methods

### Drugs preparation

GAPT, a combination of herbal extracts, was provided by Henan Wanxi Pharmaceutical Company Limited (Batch No: 20010923) and hydrochloric acid donepezil tablets were provided by Eisai (China) Pharmaceutical Company Limited (Batch No: 090508A). GAPT was dissolved in 0.5 % Carboxymethyl cellulose (CMC) at concentration of 30 mg/ml. Donepezil tablets were crashed and also dissolved in 0.5 % CMC at concentration of 0.092 mg/ml.

### Animal and administration

Three month old APPV717I mice (C57BL/6 J background strain of the transgenic mice, with mutated human APP-CT100 containing the London mutation V717I) and C57BL/6 J mice (non-transgenic inbred trains of mice, as normal control), both half male and half female, were provided by the Institute of Experimental Animals, Chinese Academy of Medical Sciences & Peking Union Medical College (Beijing, China). All animals were kept in the Pharmacological Experiment Center of Dongzhimen Hospital, Beijing University of Chinese Medicine, Beijing, PR China. They were maintained in a pathogen-free vivarium on a 12:12 h light: dark cycle (12 h light: 0600 to 1800; 12 h dark: 1800 to 0600), temperature-controlled at 24 °C and has free access to food and water. All experimental procedures with animal were performed in accordance with the National Institute of Health Guide for the Care and Use of Laboratory Animals (NIH Publications No. 80-23) revised in 1996 and had been approved by the Animal Research Ethics Board of Beijing University of Chinese Medicine.

Three-month-old male APPV717I transgenic mice were randomly divided into ten groups (*n* = 12 per group) and received intragastrically administrated vehicle or medicines: APP group was given 0.5 % CMC, Donepezil group was given donepezil (APP + D) (0.92 mg/kg/day i.g), and low dose of GAPT (APP + Gl) (0.075 g/kg/day i.g), Middle dose (APP + Gm) (0.15 g/kg/day i.g), and High dose (APP + Gh) (0.30 g/kg/day i.g) for 8 or 4 months. Three-month-old male C57BL/6 J mice as vehicle control (*n* = 12) were given 0.5 % CMC for 8 or 4 months as well.

### Immunohistochemistry and semi-quantitative analysis

All behaviorally-tested mice were deeply anesthetized by 10 % chloral hydrate (40 mg/kg body weight, i.p.), and pericardially perfused with heparinized 0.9 % saline, then removed the brain. The right hemisphere was immersion-fixed in 4 % paraformaldehyde overnight at 4 °C and then processed in phosphate buffered saline (PBS) solution containing 30 % sucrose. Seven days later, brain samples were embedded in paraffin. Serial coronal sections of the hippocampus were cut at 35 μm intervals. One of every three sections was selected and mounted onto slides for immunohistochemical staining, while the left hemisphere was snap frozen for Western blotting. Tissue from 12 rats from each group was examined.

These brain sections were deparaffinised and degraded to distilled water, then unmasked the antigen in 0.01 M Citrate Buffer with microwave, and quenched endogenous peroxidise activity by 0.3 % hydrogen peroxide in methanol for 20 min at 24 °C, then blocked in 10 % antibodies in 3 % BSA/PBS for 30 min at 37 °C. After pouring off excess serum, sections were incubated with the primary antibody in humidified boxes at 4 °C overnight. Then, sections were washed once again and incubated with biotin conjugated secondary antibodies (1:300, Fuzhou Maixin Ltd., PR China) at 37 °C for 30 min, then washed again and incubated with SABC for 1 h at 37 °C. Subsequently, sections were stained by chromogen 3’3-diaminobenzidine tetrachloride (DAB). After that sections were dehydrated, and affixed with coverslips. All brain sections chosen for staining were on a similar sagittal plane and contained approximately the same area of hippocampus. The primary antibodies used include CaMKII 1:1000 and CaN 1:100.

Average OD of each protein was measured in immunostained sections, following the instructions of the Image Pro Plus 6.0 software (Media CY Company, USA). “Nonspecific” IHC staining in sections was chosen as the control area for comparison with the immunopositive area in the neurons of the dentate gyrus. The examiner was blinded to group assignment of the samples.

### Western blotting

Western blots were performed as described previously [43]. Briefly, the snap-frozen brain tissues cut from hippocampus and cortex were weighted and homogenized with a small pestle in ice with brain tissue lysis buffer in the ratio of 1:10 (w/v) for 2 min and incubated in ice for 30 min. The homogenate was centrifuged at 13,000 r.p.m. at 4 °C for 30 min, and the supernatant was collected. Protein in the supernatant was measured by Bradford method with Coomassie Brilliant Blue G-250. Loading buffer was added to samples in the ratio of 4:1, after which they were placed in boiling water for 5 min and then chilled immediately on ice; 10 μl protein/well samples and 5 μl marker (10KD-170 KD) were loaded onto a 10 % acrylamide gel and subjected to SDS-PAGE by the Bio-Rad minigel system. Proteins were then electro-blotted onto a polyvinylidine difluoride membrane. The membrane was blocked by 5 % milk at 4 °C overnight, then incubated with the primary antibody (CaMKII 1:5000; CaN 1:4000). After three washes with PBS containing 0.5 % Tween 20, the membrane was incubated at room temperature for 1 h with HRP-conjugated secondary antibody at 1:10000 dilution on the shaker. After 3 times wash, blots were developed by the luminol reagent (Pierce Biotechnology). Densitometric analysis of the blots was completed using the Phoretix 1D software.

### Statistical analysis

All data were analyzed with SPSS 19.0 software and presented as the Mean ± SD. Comparison of different treatments was evaluated by the Student's *t* test (two-tailed). One-way ANOVA was used when comparisons were made among three groups. *P* < 0.05 was considered statistically significant.

## Results

### CaMKII and CaN expression levels in the experimental mice at the age of 7 months old

Immunohistochemistry analysis showed significant decrease of CaMKII in the CA1 region of 7 months old APPV717I transgenic mice (compare to control group *p* < 0.05), while the CaMKII expression of donepezil or GAPT treated transgenic mice were all increased, and there was significant difference between GAPT low dose treated group and the model group (*P* < 0.05). On the contrary, there was significant increase of CaN in the brain cortex of 7 months old APPV717I transgenic mice (compare to control group *p* < 0.05), and the CaN expression of donepezil or GAPT treated transgenic mice were all decreased, but there were no significant difference between each group (*P* > 0.05). Detailed data were shown in Figs. 1 and 2.

**Fig. 1:** Expression of CaMK II (Average OD) in hippocampal CA1 region in the experimental mice at the age of 7 months old were measured by immunohistochemistry staining. Note:^▲^ *p* < 0.05,vs control group, *p < 0.05,vs model group, ANOVA. CaMK II expression was determined by immunohistochemistry in the hippocampus of experimental mice. Data are expressed as mean ± SD (Average OD) of the CaMK II positive neuronal area (anti-body for CaMK II, 1:1000). Control: C57BL/6 J mice; APP: APPV717I mice; APP + D: donepezil; APP + Gl: GAPT low dose; APP + Gm: GAPT middle dose; APP + Gh: GAPT high dose

**Fig. 2:** Expression of CaN (Average OD) in hippocampal CA1 region in the experimental mice at the age of 7 months old were measured by immunohistochemistry staining. Note: ^▲^ *p* < 0.05,vs control group, ANOVA. CaN expression was determined by immunohistochemistry in the hippocampus of experimental mice. Data are expressed as mean ± SD (Average OD) of the CaN positive neuronal area (anti-body for CaN, 1:100). Control: C57BL/6 J mice; APP: APPV717I mice; APP + D: donepezil; APP + Gl: GAPT low dose; APP + Gm: GAPT middle dose; APP + Gh: GAPT high dose

Western blot analysis showed that the similar expression pattern of CaMKII and CaN in each group as immunohistochemistry analysis showed, but there was no significant difference between each group. Detailed data were shown in Fig. 3.

**Fig. 3:** Expression of CaMKII, CaN in hippocampus tissue homogenates of experimental mice at the age of 7 months were determined by western-blotting. Notes: Control: C57BL/6 J mice; APP: APPV717I mice; APP + D: donepezil; APP + Gl: GAPT low dose; APP + Gm: GAPT middle dose; APP + Gh: GAPT high dose. There was no significant difference between each group in both CaMKII, CaN

### CaMKII and CaN expression levels in the experimental mice at the age of 11 months old

Immunohistochemistry analysis showed significant decrease of CaMKII in the CA1 region of 11 months old APPV717I transgenic mice (compare to control group *p* < 0.01), while the CaMKII expression of donepezil or GAPT treated transgenic mice were all significantly increased (Donepezil vs. Model: *P* < 0.05; Gl vs. Model: *P* < 0.01; Gm vs. Model: *P* < 0.01; Gh vs. Model: *P* < 0.05), and the GAPT low dose treated group had the highest CaMKII expression level. Detailed data were shown in Fig. 4. There was significant increase of CaN in the CA1 region of 11 months old APPV717I transgenic mice (compare to control group *p* < 0.01), while the CaN expression of donepezil or GAPT treated transgenic mice were all decreased, and there were significant differences between donepezil or GAPT high dose treated transgenic mice group and model group (Donepezil vs. Model: *P* < 0.05;Gh vs. Model: *P* < 0.05), and the GAPT high dose treated group had the lowest CaN expression level. Detailed data were shown in Figs. 4 and 5.

**Fig. 4:** Expression of CaMKII (Average OD) in hippocampal CA1 region in the experimental mice at the age of 11 months old were measured by immunohistochemistry staining. Notes:^▲^ *p* < 0.05, ^▲▲^ *p* < 0.01,vs control group, *p < 0.05, **p < 0.01,vs model group, ANOVA. Control: C57BL/6 J mice; APP: APPV717I mice; APP + D: donepezil; APP + Gl: GAPT low dose; APP + Gm: GAPT middle dose; APP + Gh: GAPT high dose. CaMKII expression was determined by immunohistochemistry in the hippocampus of experimental mice. Data are expressed as mean ± SD (Average OD) of the CaMKII positive neuronal area (anti-body for CaMKII, 1:1000)

**Fig. 5:** Expression of CaN (Average OD) in hippocampal CA1 region in the experimental mice at the age of 11 months old were measured by immunohistochemistry staining. Notes:^▲^ *P* < 0.05, ^▲▲^ *P* < 0.01, vs Control group, *P < 0.05,vs model group, ANOVA. Control: C57BL/6 J mice; APP: APPV717I mice; APP + D: donepezil; APP + Gl: GAPT low dose; APP + Gm: GAPT middle dose; APP + Gh: GAPT high dose. CaN expression was determined by immunohistochemistry in the hippocampus of experimental mice. Data are expressed as mean ± SD (Average OD) of the CaN positive neuronal area (anti-body for CaN, 1:100)

Western blot analysis showed that the similar expression pattern of CaMKII and CaN in each group as immunohistochemistry analysis showed, but there was no significant difference in the expression of CaMKII and CaN between each group. Detailed data were shown in Fig. 6.

**Fig. 6:** Expression of CaMKII, CaN in hippocampus tissue homogenates of experimental mice at the age of 11 months were determined by western-blotting. Notes: Control: C57BL/6 J mice; APP: APPV717I mice; D: donepezil; Gl: GAPT low dose; APP + Gm: GAPT middle dose; APP + Gh: GAPT high dose. There was no significant difference in the expression of CaMKII and CaN between each group

## Discussion

APP/V717I transgenic mice used in this study were of the C57BL/6 J genetic background and carrying mutated human APP-CT100 containing the London mutation *V717I*, which is characterized by the increased generation of Aβ_42_ and AD-like pathological changes [46]. However, the formation of amyloid plaques in the mice only initiates around their 9 months old [47, 48], and which is preceded by earlier phenotypic changes that comprise impaired LTP and cognitive defects as early as age 4–6 months [49]. These findings indicate the critical involvement of amyloid peptides in defective LTP of APP transgenic mice. But the mechanisms behind the defective LTP in this transgenic mouse are still not clear. Especially, the expression of CaMKII and CaN in the brain of this transgenic mouse are not well investigated. In order to observe levels of CaMKII and CaN before and after amyloid plaques formation, as well as to reveal whether the cognitive improving effects of GAPT is conducted through rebalance CaMKII and CaN, APPV717I transgenic mice aged 3 months were used in our experiment and treated with GAPT up to their 7 or 11 months. That is 3 months old APPV717I transgenic mice were treated by GAPT extracts for 4 months or 8 months in this study.

GAPT, also called GEPT in our previous papers, is a combination of eight herbal extracts. It has showed marked enhancement to the function of learning and memory of AD rat model induced by Aβ_1-42_peptide, as well as APPV717I transgenic mice during the 8 months’ treatment [43, 44]. It's reduction of endogenous Aβ peptide in the brain of APPV717I transgenic mice may conducted via the inhibition of PS1 activity rather than BACE1, as well as the promotion of insulin-degrading enzyme (IDE) and neprilysin activity [43]. And previous preliminary clinical study also indicated that a three month treatment of GAPT had significant effectiveness in improving memory and cognitive impairment and delaying memory decline through one year in 70 patients with aMCI [50]. However, it is unknown for mechanisms behind synaptic protection effects of GAPT in APPV717I transgenic mice. Spatial learning and memory ability of all mice were measured by Orientation Navigation Tests and Spatial Probe Tests with Morris Water Maze (MWM), which found that GAPT significantly improve the spatial learning and memory of APPV717I transgenic mice during the 8 months’ treatment (detailed data will be published in another article).

Immunohistochemistry analysis showed that there were significant decrease of CaMKII expression in the CA1 region of APPV717I transgenic mice, while the CaMKII expression of donepezil or GAPT treated transgenic mice were increased. Although there was only significant difference between GAPT low dose treated group and the model group in 7 months old mice, there were significant differences between each treated group and the model group in 11 months old mice, and the GAPT low dose treated group had the highest CaMKII expression level. Thus, the CaMKII expression is gradually decreased in the brain of APPV717I transgenic mice, and the increase effects of donepezil or GAPT on CaMKII expression is time-dependent. The longer treatment the better increase effects.

Immunohistochemistry analysis showed significant increase of CaN in the brain cortex of APPV717I transgenic mice, and there were decrease in CaN expression in donepezil or GAPT treated transgenic group. However, there were only significant differences between donepezil or GAPT high dose treated transgenic mice group and model group in 11 months old mice, and the GAPT high dose treated group had the lowest CaN expression level. The present result shows that the CaN expression is gradually increased in the brain of APPV717I transgenic mice,and the decrease effects of donepezil or GAPT on CaMKII expression is also time-dependent.

These results were consistent with others researches. For example, it has been shown that there was reduced p-CaMKII level in specific brain regions in AD patients, such as frontal cortex and hippocampus [51] and there were decreased CaMKII activation and increased CaN levels in a short-term memory and E-LTP deficits rat model induced by beta amyloid and stress [52]. These kinds of changes also have been shown to contribute to the inhibition of LTP in CA1 region or dentate gyrus of rat hippocampus by acute application of synthetic beta amyloid. And such inhibition of LTP can be blocked by specific inhibitors of CaN [53, 54].

Western blot analysis showed the similar expression pattern of CaMKII and CaN in each group in 7 or 11 months old mice as immunohistochemistry analysis showed, but there was no significant difference between each group. This may partially because there are different expression levels of CaMKII and CaN in different cells, and there are different status of those two proteins, active or inactive. For example, there are evidences suggest that Aβ induces different changes of CaN expression in neurons and astrocytes, and CaN A, the catalytic subunit of CaN, is proteolytically activated in AD cortex by the degradation of an autoinhibitory domain [39, 40] and which is expressed in reactive astrocytes surrounding senile plaques [41]. As far as CaMKII expression is concerned, very early research has found no alteration of CaMKII expression in the AD brain [55], and only recent research has found phosphorylated CaMKII expression was reduced in the frontal cortex and hippocampus of AD brains [51]. Therefore, further studies about specific status of those two proteins in certain brain cells of the APPV717I transgenic mice are needed.

However, these data is fully valid to indicate that GAPT extract may balance the expression of CaMKII and CaN in the brain of APPV717I transgenic mice. And different doses of GAPT may have slight difference in the influence of those two proteins. That is, high dose GAPT have potentially higher CaN inhibiting effects, while low dose may have higher CaMKII activating effects in APP mice. And all these effects can be exerted before the formation of amyloid plaques. This may partially explain the A 24-week preliminary study of GAPT showed a significant improvement on cognitive function in patients with aMCI, an early stage of AD [45, 56].

## Conclusion

There were obvious disturbance of CaMKII and CaN expression in the CA1 region of APPV717I transgenic mice either before or after the formation of amyloid plaques. While, GAPT extract have significant effectiveness in restoring the balance of CaMKII and CaN, that is activating the expression of CaMKII and inhibiting the expression of CaN. This may partially explain the cognitive improving effects of GAPT in APPV717I transgenic mice.

## Abbreviations

AD, Alzheimer's disease; aMCI, amnestic mild cognitive impairment; AMPAR, α-amino-3-hydroxy-5-methyl-4-isoxazolepropionic acid receptor; Aβ, amyloid beta; CaMKII, Ca2+/calmodulin (CaM)-dependent protein kinase II; CaN. Ca2+/Calmodulin-dependent protein phosphatase 2B or calcineurin; CMC, Carboxymethyl cellulose; DAB, 3’3-diaminobenzidine tetrachloride; IDE, insulin-degrading enzyme; IHC, immunohistochemical; LTP, long-term potentiation; MWM, Morris Water Maze; PBS, phosphate buffered saline; PP1, protein phosphatase 1; PP2B, protein phosphatase 2B

## References

[1] Reitz C, Brayne C, Mayeux R (2011). Epidemiology of Alzheimer disease. Nat Rev Neurol.

[2] Davies CA, Mann DMA, Sumpter PQ, Yates PO (1987). A quantitative morphometric analysis of the neuronal and synaptic content of the frontal and temporal cortex in patients with Alzheimer's disease. J Neurol Sci.

[3] Blennow K, Bogdanovic N, Alafuzoff I, Ekman R, Davidsson P (1996). Synaptic pathology in Alzheimer's disease: Relation to severity of dementia, but not to senile plaques, neurofibrillary tangles, or the ApoE4 allele. J Neural Transm.

[4] Ingelsson M, Fukumoto H, Newell KL, Growdon JH, Hedley-Whyte ET, Frosch MP, Albert MS, Hyman BT, Irizarry MC (2004). Early Abeta accumulation and progressive synaptic loss, gliosis, and tangle formation in AD brain. Neurology.

[5] Bliss TVP, Collingridge GL (1993). A synaptic model of memory: long-term potentiation in the hippocampus. Nature.

[6] Kennedy MB (1989). Regulation of synaptic transmission in the central nervous system: Long-term potentiation. Cell.

[7] Nicoll RA, Malenka RC (1995). Contrasting properties of two forms of long-term potentiation in the hippocampus. Nature.

[8] Stevens CF (1998). A million dollar question: Does LTP = Memory?. Neuron.

[9] Lisman J, Schulman H, Cline H (2002). The molecular basis of CaMKII function in synaptic and behavioural memory. Nat Rev Neurosci.

[10] Silva A, Stevens C, Tonegawa S, Wang Y (1992). Deficient hippocampal long-term potentiation in alpha-calcium-calmodulin kinase II mutant mice. Science.

[11] Soderling TR (1993). Calcium/calmodulin-dependent protein kinase II: role in learning and memory. Mol Cell Biochem.

[12] Griffith LC (2004). Calcium/Calmodulin-dependent protein Kinase II: an unforgettable Kinase. J Neurosci.

[13] Stevens CF, Tonegawa S, Wang Y (1994). The role of calcium calmodulin kinase II in three forms of synaptic plasticity. Curr Biol.

[14] Mansuy IM (2003). Calcineurin in memory and bidirectional plasticity. Biochem Biophys Res Commun.

[15] Hara MR, Snyder SH (2007). Cell signaling and neuronal death. Annu Rev Pharmacol Toxicol.

[16] Kennedy MB, Bennett MK, Bulleit RF, Erondu NE, Jennings VR, Miller SG, Molloy SS, Patton BL, Schenker LJ (1990). Structure and regulation of type II calcium/calmodulin-dependent protein kinase in central nervous system neurons. Cold Spring Harb Symp Quant Biol.

[17] Anderson M, Braun A, Schulman H, Premack B (1994). Multifunctional Ca2+/calmodulin-dependent protein kinase mediates Ca(2+)-induced enhancement of the L-type Ca2+ current in rabbit ventricular myocytes. Circ Res.

[18] Neal Waxham M, Malenka RC, Kelly PT, Mauk MD (1993). Calcium/calmodulin-dependent protein kinase II regulates hippocampal synaptic transmission. Brain Res.

[19] Ouimet CC, McGuinness TL, Greengard P (1984). Immunocytochemical localization of calcium/calmodulin-dependent protein kinase II in rat brain. Proc Natl Acad Sci U S A.

[20] Erondu NE, Kennedy MB (1985). Regional distribution of type II Ca2+/calmodulin-dependent protein kinase in rat brain. J Neurosci.

[21] Fukunaga K, Goto S, Miyamoto E (1988). Immunohistochemical localization of Ca2+/Calmodulin-dependent protein Kinase II in Rat brain and various tissues. J Neurochem.

[22] Peng J, Kim MJ, Cheng D, Duong DM, Gygi SP, Sheng M (2004). Semiquantitative proteomic analysis of rat forebrain postsynaptic density fractions by mass spectrometry. J Biol Chem.

[23] Rich DP, Cdlbran RJ, Schworer CM, Soderling TR (1989). Regulatory properties of calcium/calmodulin-dependent protein Kinase II in rat brain postsynaptic densities. J Neurochem.

[24] Fukunaga K, Stoppini L, Miyamoto E, Muller D (1993). Long-term potentiation is associated with an increased activity of Ca2+/calmodulin-dependent protein kinase II. J Biol Chem.

[25] Ito I, Hidaka H, Sugiyama H. Effects of KN-62, a specific inhibitor of calcium/calmodulin-dependent protein kinase II, on long-term potentiation in the rat hippocampus. Neurosci Lett. 1991;121(1–2):119–21.10.1016/0304-3940(91)90663-e1850502

[26] Malinow R, Schulman H, Tsien R (1989). Inhibition of postsynaptic PKC or CaMKII blocks induction but not expression of LTP. Science.

[27] Silva A, Paylor R, Wehner J, Tonegawa S (1992). Impaired spatial learning in alpha-calcium-calmodulin kinase II mutant mice. Science.

[28] Shirke AM, Malinow R (1997). Mechanisms of potentiation by calcium-calmodulin kinase ii of postsynaptic sensitivity in rat hippocampal CA1 Neurons. J Neurophysiol.

[29] Lledo PM, Hjelmstad GO, Mukherji S, Soderling TR, Malenka RC, Nicoll RA (1995). Calcium/calmodulin-dependent kinase II and long-term potentiation enhance synaptic transmission by the same mechanism. Proc Natl Acad Sci.

[30] Poncer JC, Esteban JA, Malinow R (2002). Multiple Mechanisms for the potentiation of AMPA receptor-mediated transmission by α-ca2+/calmodulin-dependent protein kinase II. J Neurosci.

[31] Matsui H, Itano T, Etoh S, Tokuda M, Wang JH, Hatase O (1989). Demonstration of different regional distributions of calcineurin subunits using monoclonal antibodies. Adv Exp Med Biol.

[32] Foster TC, Sharrow KM, Masse JR, Norris CM, Kumar A (2001). Calcineurin links Ca2+ dysregulation with brain aging. J Neurosci.

[33] Dineley KT, Hogan D, Zhang W-R, Taglialatela G (2007). Acute inhibition of calcineurin restores associative learning and memory in Tg2576 APP transgenic mice. Neurobiol Learn Mem.

[34] Zeng H, Chattarji S, Barbarosie M, Rondi-Reig L, Philpot BD, Miyakawa T, Bear MF, Tonegawa S (2001). Forebrain-specific calcineurin knockout selectively impairs bidirectional synaptic plasticity and working/episodic-like memory. Cell.

[35] Taglialatela G, Hogan D, Zhang W-R, Dineley KT (2009). Intermediate- and long-term recognition memory deficits in Tg2576 mice are reversed with acute calcineurin inhibition. Behav Brain Res.

[36] Malleret G, Haditsch U, Genoux D, Jones MW, Bliss TVP, Vanhoose AM, Weitlauf C, Kandel ER, Winder DG, Mansuy IM (2001). Inducible and reversible enhancement of learning, memory, and long-term potentiation by genetic inhibition of calcineurin. Cell.

[37] Lian Q, Ladner CJ, Magnuson D, Lee JM (2001). Selective changes of calcineurin (protein phosphatase 2b) activity in Alzheimer's disease cerebral cortex. Exp Neurol.

[38] Ladner CJ, Czech J, Maurice J, Lorens SA, Lee JM (1996). Reduction of calcineurin enzymatic activity in Alzheimer's disease: correlation with neuropathologic changes. J Neuropathol Exp Neurol.

[39] Celsi F, Svedberg M, Unger C, Cotman CW, Carrì MT, Ottersen OP, Nordberg A, Torp R (2007). Beta-amyloid causes downregulation of calcineurin in neurons through induction of oxidative stress. Neurobiol Dis.

[40] Liu F, Grundke-Iqbal I, Iqbal K, Oda Y, Tomizawa K, Gong CX (2005). Truncation and activation of calcineurin a by calpain i in alzheimer disease brain. J Biol Chem.

[41] Norris CM, Kadish I, Blalock EM, Chen KC, Thibault V, Porter NM, Landfield PW, Kraner SD (2005). Calcineurin triggers reactive/inflammatory processes in astrocytes and is upregulated in aging and Alzheimer's models. J Neurosci.

[42] Yamin G (2009). NMDA receptor-dependent signaling pathways that underlie amyloid β-protein disruption of LTP in the hippocampus. J Neurosci Res.

[43] Tian J, Shi J, Zhang L, Yin J, Hu Q, Xu Y, Wang R, et al. GEPT extract reduces Abeta deposition by regulating the balance between production and degradation of Abeta in APPV717I transgenic mice. Curr Alzheimer Res. 2009;6(2):118–31.10.2174/15672050978760294219355846

[44] Tian J, Xu Y, Sheng S, Shi J, Yin J, Wang Y (2006). Influence of GETO extract on myelin sheath structure and myelin basic protein content in the brain with AD model. Alzheimers Dement.

[45] Miao Y (2008). Part 5: a randomized, double-blind and parallel control study of GEPT extract in the treatment of amnestic mild cognitive impairment.

[46] Sturchler-Pierrat C, Abramowski D, Duke M, Wiederhold K-H, Mistl C, Rothacher S, et al. Two amyloid precursor protein transgenic mouse models with Alzheimer disease-like pathology. Proc Natl Acad Sci U S A. 1997;94(24):13287–92.10.1073/pnas.94.24.13287PMC243019371838

[47] Dewachter I, Van Dorpe J, Smeijers L, Gilis M, Kuiperi C, Laenen I, Caluwaerts N, Moechars D, Checler F, Vanderstichele H (2000). Aging increased amyloid peptide and caused amyloid plaques in brain of old app/v717i transgenic mice by a different mechanism than mutant presenilin1. J Neurosci.

[48] Johnson-Wood K, Lee M, Motter R, Hu K, Gordon G, Barbour R, Khan K, Gordon M, Tan H, Games D (1997). Amyloid precursor protein processing and Aβ42 deposition in a transgenic mouse model of Alzheimer disease. Proc Natl Acad Sci U S A.

[49] Dewachter I, Reversé D, Caluwaerts N, Ris L, Kuipéri C, Van den Haute C, Spittaels K, Umans L, Serneels L, Thiry E (2002). Neuronal deficiency of presenilin 1 inhibits amyloid plaque formation and corrects hippocampal long-term potentiation but not a cognitive defect of amyloid precursor protein [V717I] transgenic mice. J Neurosci.

[50] Tian J, Zhu AH, Zhong J (2003). The effectiveness of GETO in the treatment of mild cognitive impairment in community elderly, A follow-up study on a randomized, single-blind control of GETO pills in treatment of memory disorder in elderly people with MCI in a Beijing community. [Article in Chinese]. Zhongguo Zhong Yao Za Zhi.

[51] Amada N, Aihara K, Ravid R, Horie M (2005). Reduction of NR1 and phosphorylated Ca2+/calmodulin-dependent protein kinase II levels in Alzheimer's disease. Neuroreport.

[52] Srivareerat M, Tran TT, Alzoubi KH, Alkadhi KA (2009). Chronic psychosocial stress exacerbates impairment of cognition and long-term potentiation in β-amyloid rat model of Alzheimer’s disease. Biol Psychiatry.

[53] Chen Q-S, Wei W-Z, Shimahara T, Xie C-W (2002). Alzheimer amyloid [beta]-peptide inhibits the late phase of long-term potentiation through calcineurin-dependent mechanisms in the hippocampal dentate gyrus. Neurobiol Learn Mem.

[54] Zhao D, Watson JB, Xie CW (2004). Amyloid β prevents activation of calcium/calmodulin-dependent protein kinase ii and ampa receptor phosphorylation during hippocampal long-term potentiation. J Neurophysiol.

[55] Simonian NA, Elvhage T, Czernik AJ, Greengard P, Hyman BT (1994). Calcium/calmodulin-dependent protein kinase II immunostaining is preserved in Alzheimer's disease hippocampal neurons. Brain Res.

[56] Tian J, Shi J, Zhang X, Wang Y (2010). Herbal therapy: a new pathway for the treatment of Alzheimer's disease. Alzheimers Res Ther.

